# Analysis of Chinese Painting Color Teaching Based on Intelligent Image Color Processing Technology in the Network as a Green Environment

**DOI:** 10.1155/2022/8303496

**Published:** 2022-06-21

**Authors:** Li Tian

**Affiliations:** Zhengzhou Normal University, Zhengzhou, Henan 450000, China

## Abstract

This work was conducted to study the Chinese painting color teaching analysis of intelligent image color processing technology under the network environment. First, the paper preprocesses the obtained color mural images, realizes the automatic recognition and marking of the images with different defect degrees and color fading, and uses denoising and texture background elimination to remove unnecessary background information. Then, according to the characteristic that the repair order of boundary points in the Criminisi algorithm is determined by the size of priority weight, the data items and confidence items are added. Finally, the design uses image processing technology and the loss formula to identify the connecting edge of the color area to be taught, establish the color extraction area, calculate the bit weight of the best color, find out the color extraction position, and synthesize different colors according to the original painting color superposition method. The partial differential equation is used to set the teaching code of color teaching system to realize the teaching of Chinese painting color. The experimental results show that compared with the original teaching system, the designed color teaching system has a stronger ability to recognize the edge of Chinese painting color teaching, and the quality of Chinese painting after teaching is higher. It can be seen that the color teaching system can be applied to the color teaching of Chinese painting.

## 1. Introduction

Digital image processing is a relatively young subject compared with the history of human fascination with visual mechanism. However, in its short history, it has been applied to almost all fields related to imaging with varying degrees of success. In recent years, the field of digital image processing has developed rapidly. Digital image has become an effective tool for scholars in psychology, physiology, computer science, and many other fields to study visual perception. The demand for image processing in military, remote sensing, meteorology, and other large-scale applications is also growing. With the development and popularization of multimedia technology, digital image processing technology and video technology have changed from professional terms to people's daily language. As a traditional painting with a long history and fine tradition, Chinese painting condenses a large amount of historical information of the Chinese nation and embodies the national wisdom of generations of people and the character of each period. At the same time, it also reflects the historical development trend, the state power reform, and other social development [1]. It can be seen that Chinese painting is not only the embodiment of China's 5000-year national spirit but also fully reflects the historical development process of the country. However, because Chinese painting appeared early and spread for a long time, it led to local fading, edge fading, and overall halo in the original colorful and bright Chinese painting. In the teaching process of Chinese painting major, color teaching is one of the compulsory courses. Quality education requires students not only to understand and master professional knowledge and skills but also to improve their comprehensive quality in the learning process and promote their all-round development. In Chinese painting color teaching, how to effectively convey the spiritual connotation of Chinese painting color to students is very important. The study of the color connotation of Chinese painting can not only help students master painting skills but also effectively cultivate students' comprehensive quality and promote students' all-round development.

Because of the rapid development of modern computer technology and image processing technology, the color teaching of mural cultural relics has become simple and fast. Digital image processing has been widely used in the early 20th century and has gradually become a hot subject. Based on the mathematical algorithm, this technology can improve the image quality and modify the image (Figure 1) and can also extract effective information from the image to make the image effect more in line with the visual requirements of human eyes. In addition, digital image processing technology plays an important role in the virtual restoration, reproduction, and evolution simulation of traditional Chinese painting [2].

Therefore, a color teaching system of Chinese painting is designed. Through this system, the teaching area and teaching location nodes are set to teach the painting with fading problems. However, the faded edge of Chinese painting taught by this system is inconsistent with the teaching edge, resulting in an obvious edge contour color in the painting. Therefore, aiming at this problem of the original teaching system, a new Chinese painting color teaching system is designed based on image processing technology. The system focuses on the recognition ability of teaching edge to ensure that there is no color difference between the edge color and the natural color of painting [3]. The emergence of Chinese painting color teaching system has improved the teaching ability of Chinese painting color, strengthened the protection of painting, continued the Chinese painting with stories and ideas, and provided technical support for painting color teaching in other countries.

This study develops a color identification mode under the network environment, which can promote the online (rather than offline) image processing and creation and contribute to the environmental protection and energy saving by no waste of paper and painting materials.

## 2. Literature Review

Teixeira et al. first proposed the hierarchical transformation of digital images and finally used the hierarchical fusion mechanism to find the best teaching relationship between each layer, so that the traditional Chinese painting after teaching achieves a good visual effect [4]. Han et al. used the halftone processing mechanism of the image to obtain effective prior knowledge to restore the image, which effectively improves the teaching quality of the image [5]. Then, Liu et al. proposed a fast optimization transfer algorithm (FOTA) based on the overall variational model, which changed the univariate function into the bivariate function and improved the teaching efficiency. However, when these model algorithms are used to teach a large area of missing image information or some images with texture, the effect is fuzzy and the image edge features are poor. Moreover, the above algorithms restore the image according to the characteristics of the known pixels in the surrounding pixels and damaged edge areas, ignoring the high-frequency components of the image [6]. In recent years, many scholars have improved image teaching algorithms to improve the image effect and quality, so as to meet the vision of human eyes. Hsing Yu et al. combined the partial differential equation with the sample and used the Euler equation of global variation combined with the original data item function to determine the order of sample block teaching, so as to teach the image [7]. Melekhin et al. took the D-S evidence theory as the confidence term and combined it with a TV model as the priority function. The algorithm effectively uses the image structure and texture information and obtains a better teaching effect [8]. Xing et al. added the image segmentation theory to the image teaching algorithm, reduced the search area to some relevant information areas, reduced the search scope while ensuring the teaching quality, and improved the teaching method. However, these algorithms need a long process in time, which is not conducive to rapid teaching [9]. Duan et al. summarized the impact of different acquisition technologies and methods on cultural relic images and digital protection. Through the analysis and summary of existing optical measurement instruments, measurement technologies, and sensors, accurate teaching data were obtained [10]. Singh et al., combining with the method of chemical analysis, proposed a method of preferentially repairing the gradient to carry out virtual teaching of ancient traditional Chinese painting, transfer the gradient of the known area of the image to the damaged area, and make the image model more optimized [11]. Liu et al. optimized the matching target criterion used in the algorithm, proposed the color gradient method for block matching, deduced the teaching method of gray image, and achieved a certain teaching effect [12].

## 3. Method

### 3.1. Digital Image Teaching Technology Based on Sample Texture

Computer graphics is a new subject that studies how to generate, process, and display graphics with digital computer. It focuses on how to turn data and geometric models into images, which corresponds to another technology: pattern recognition. Pattern recognition focuses on how to extract data and models from images, which are the opposite process. In addition, there is another discipline specialized in the geometric model and data processing, which is computing. It focuses on the computer representation and analysis and synthesis of geometric objects and studies how to establish the mathematical model of geometric objects conveniently and flexibly, how to improve the efficiency of algorithm, and how to better store and manage these model data in the computer [13]. At present, the most active research of computational geometry can be the construction and splicing of curves and surfaces, three-dimensional modeling, scattered data interpolation, computational complexity, and so on. The relationship of all related technologies is shown in Figure 2.

The purpose of digital image teaching is to fill the defect information in the image through a system, restore the original appearance of the image, and meet the aesthetic requirements of human vision, so that the observer will not notice that the image has been damaged or taught before. The general image processing model is represented as the input-output system shown in Figure 3.

In the basic model of image processing, U1 is an image or a series of images, the image processing system is a linear or nonlinear processing algorithm, such as denoising, restoration, coding, and compression, and U2 is the output characteristic image.

Image teaching needs to emphasize the coherence and structural integrity of the texture in the defect area. Therefore, when using the sample-based texture synthesis technology in image teaching, it is necessary to adopt a strategy different from the previous texture synthesis.

First, texture synthesis technology generally adopts the scanning sequence from top to bottom to left and right or spiral to synthesize regular new textures [14]. The teaching area of the image is often very irregular, so it should be processed layer-by-layer from the periphery to the interior of the teaching area, and it is not suitable to adopt a fixed processing order for texture synthesis. Second, in the process of teaching the specific damaged natural image, according to the direction of the structural line around the area to be taught, extend the structural line and connect it to the inside of the area to be taught, while taking into account the continuity of the structural line along the edge of the damaged area and the maintenance of the texture detail content, search the matching block along the structural line direction of the known area, and copy the found matching texture detail module to the damaged area. Suppose the digital model of simplified image teaching is as shown in Figure 4: let *I* represent the damaged image to be taught and Φ is the information defect part in image *I*. The whole process of image teaching is to judge and guess according to the effective information in the known area Φ under the condition of meeting the requirements of human vision, fill in the information of the area to be taught Φ, and finally teach as a complete image.

The specific steps of the sample-based image teaching algorithm are as follows: first, calculate the priority value of each point of the filling boundary of the damaged area by using the following equation:

(1) $$\begin{array}{c} P\left(p\right)=C\left(p\right)D\left(p\right), \end{array}$$

where

(2) $$\begin{array}{c} C\left(p\right)=\frac{\sum C\left(q\right)}{\left|\psi_{p}\right|}, \end{array}$$

(3) $$\begin{array}{c} D\left(p\right)=\frac{\left|\nabla I_{p}\cdot n_{p}\right|}{\alpha }. \end{array}$$

Among them, *C*(*p*) is called the confidence term of the block to be taught and expressed as the proportion of effective pixels in the block to be taught, and it represents the amount of effective information around a pixel *p*. *D*(*p*) is the data item of the block to be taught, *n*_*p*_ is the unit normal vector of the contour at point *p*, Δ_*p*_^*I*^ is the isoilluminance perpendicular to the gradient of point *p*, and the initialization of *C*(*p*) is

(4) $$\begin{array}{c} C\left(p\right)=\left\{\begin{array}{c} 0,p\in D\\ 1,p\in \left(\Omega /D\right) \end{array}\right\}. \end{array}$$

The Criminisi algorithm takes the repair order of boundary points as the center, first finds the optimal value, and then finds the best sample block. Matching according to the similarity between the area to be repaired and the optimal sample block makes the ductility of image structure and texture look more natural after teaching. However, when searching by pixel, if the edge information of the image is ignored, the method of calculating priority weight only includes the boundary features around the repaired area [15], error accumulation and fuzziness will occur. After each priority calculation, when updating the priority of all sample blocks on the leading edge of image filling, the confidence of damaged pixels in the image to be taught should be updated to equation (5) to reduce the change trend of gradual reduction of partial confidence.

(5) $$\begin{array}{c} C^{\prime }\left(p\right)=\frac{\sum C\left(p\right)}{\left|\psi_{p}\right|}. \end{array}$$

Error accumulation will occur when the Criminisi algorithm directly updates the confidence.  Figure 5(a) is the original image, Figure 5(b) is the target area mark, and Figure 5(c) is the teaching effect diagram of optimizing the processing of strong edge information areas. It can be seen from the renderings in Figures 5(a) and 5(c) that the effect of continuous optimization of strong edges is not very good. This is mainly because in this algorithm, the priority is calculated by *P*(*p*)=*C*(*p*)*D*(*p*). If the confidence term *C*(*p*) is equal, the greater the *D*(*p*), the higher the priority, and the priority of the block where the strong edge is located will be higher than that of other data blocks. However, there will be bad effects in the process of processing. Here, curvature can be added to the priority to change the priority size, avoid the error of filling order, and alleviate the error accumulation.

In practical application, the effect of this algorithm is not so ideal. It only performs matching search in the specified effective area. The disadvantage of using the global search mode to search the matching sample block is low efficiency, and the size of the template will have a great impact on the search and filling. In addition, finding the matching block takes a long time, high cost, and low efficiency. In the process of filling the image with the sample texture algorithm [16], with the increase of the number of iterations, the confidence item will quickly drop to zero. Even if the data item is large, the priority function will gradually become zero, resulting in inaccurate teaching sequence and image teaching distortion and affecting the teaching effect. Therefore, the priority function is changed to

(6) $$\begin{array}{c} P\left(p\right)=\left(1-\lambda \right)e^{C\left(p\right)}+\lambda D\left(p\right),\left(0<\lambda <1\right), \end{array}$$

where *λ* is the weight coefficient, and in the original priority mathematical model, the confidence item and the data item are replaced by the additive form. The weights of *C*(*p*) and *D*(*p*) are changed by adjusting the value of the brother, that is to say, the weights of the structural information and texture information in the priority calculation process are adjusted in the process of digital mural image restoration. Through the comparison of experiments and relevant literature, it is found that when the value of brother is up and down in the range of 0.38, the processed image signal-to-noise ratio is better and the time optimization is better.

### 3.2. Color Region Extraction Technology of Color Table Clustering

In the image database, the image objects distributed in the image have different positions, sizes, and orientations, and the starting points of these shape boundaries are also different in the process of extracting shape boundaries. Therefore, these situations need to be standardized to make the shape description in a unified coordinate position, unified size, unified orientation, and unified starting point, so as to ensure that the shape description is independent of the spatial orientation of the shape. We use the regional features of shapes to normalize them. The specific process is shown in Figure 6.

At first, we get the center of gravity (*x*_*c*_, *y*_*c*_) of the image object and then translate the center of gravity of the image object to the coordinate origin, so as to ensure that all shapes are independent of their specific positions in the image. Generally speaking, for a shape, its principal axis is unique (except for shapes such as polygons and circles), so the direction of its principal axis can be used to represent the direction of the whole object. Because different objects have different directions, the principal axis of each object can be rotated to coincide with the *x*-axis or *y*-axis, so as to ensure that different image objects have a unified orientation. For different images, the size of the object is different. We define the radius of the shape as the maximum distance from all boundary points of the shape to its center of gravity. It can be seen that for a specific shape [17], its radius is certain. We can uniformly shrink the whole shape with the center of gravity as the scaling center, so that these shapes can be compared in a unified size. Then, the object is transformed symmetrically along the *x*-axis or *y*-axis. This process is called the normalization of shape objects.

#### 3.2.1. Color Image Adaptive Threshold Processing

The purpose of threshold processing is to segment the image, remove the multicolor background from the object, and fill it with white, so that the background of the image is relatively single, which is conducive to the subsequent color histogram analysis, as shown in Figure 7.

#### 3.2.2. Histogram Analysis of Color Frequency

1. The color frequency histogram of the image after the threshold is calculated.
2. According to the Euclidean distance of space of two colors, the similarity clustering of color frequency histogram is carried out: the nearest neighbor principle is adopted to merge the close color classes in the color table.
3. The color frequency histogram is sorted according to the frequency, and the direction is from large to small.
4. According to the color table and color frequency histogram, the average value of the colors contained in the color class is obtained, and this average value is taken as the typical color of this class. The white background has the largest value in frequency, which is helpful to distinguish the background from the target color class.

#### 3.2.3. Color Clustering

If a color is closest to the color in the cluster, it will be clustered into that category. The clustering results show the hierarchical results in the form of multiple windows. The key algorithms are as follows:

1. The algorithm for determining the color separation number: when the user gives the merging color difference, the computer merges the colors. When merging is impossible, the remaining color number is the color separation number.
2. The spot color separation color selection algorithm: transform many colors into several colors and make the changed image have the minimum color difference.
3. The image color separation processing algorithm (no jitter and jitter).
4. The color points of color separation are omitted.

### 3.3. Knowledge Expression of Mural Images

We call semantic features such as image content and background and experts' empirical knowledge and experimental statistical knowledge as knowledge. The knowledge referred to here is actually a kind of domain knowledge [18]. In the field of traditional Chinese painting, the knowledge mainly includes the following:

1. The experience and knowledge accumulated by artists for a long time: this kind of knowledge is usually summarized on the basis of referring to historical documents and relevant pictures and researching the clothing system, bun decoration, and customs, which has universal guiding significance.
2. Traditional Chinese painting protects the knowledge of scientists: this kind of knowledge is the discoloration mechanism of pigments obtained through the analysis of pigment chemical experiments. This kind of knowledge accurately reflects the discoloration law of lead containing pigments. For example, lead (pb304) changes from orange red to brown red and finally black red under the sun.
3. From the mural's own knowledge: because of the long history, the change of environmental conditions, and other objective reasons, it is impossible to comprehensively and accurately grasp the chemical change law of the pigments of different components of traditional Chinese painting and the color assignment method of traditional Chinese painting. Therefore, the mural itself plays a particularly prominent role as a source of knowledge. Here, it refers to works that do not change color or do not change color seriously.
4. Experimental knowledge obtained from the computer simulation test: because there are some special cases, there is no ready-made above two kinds of knowledge as a reference. At this time, we use the characteristics of computer easy test to test a variety of restoration functions and select the restoration function that is most likely to meet the actual situation as a special empirical knowledge according to its effect.

Traditional Chinese painting is the same to the above painting styles, and each mural was painted in a specific dynasty and a specific cave at that time. Therefore, we believe that the investigation of traditional Chinese painting can be carried out from the three dimensions of time, space, and style, as shown in Figure 8, which provides a basis for the design of mural library. At present, the investigation of traditional Chinese painting mainly studies the development and evolution process of mural style from the time dimension, while the space dimension mainly represents the specific location of the hole window wall of a mural, which is not the key of the research [19].

The evolution process of discoloration and fading is a color transition process. Color transition refers to finding a transition curve in the color space to slowly change from one color to another [20]. Considering that the discoloration or the fading process usually starts relatively fast and then slows down slowly, it is not appropriate to adopt linear transition. There are two ways to achieve this effect: one is to insert intermediate color transition values and use these transition values to control the evolution speed, and from these transition values, a Bessel curve can be obtained as the transition curve of color transition; the second method is to use some nonlinear functions. At first, the slope is relatively large and then gradually slows down.

In fact, the intermediate process of transferring from one color to another with constraints is in line with the color transition. We can get several typical intermediate colors by setting the specific values of transparency and white matter ratio at typical times and using the computer color mixing model. However, the discoloration and fading of pigment is a relatively continuous track, which requires us to use the typical intermediate color simulation to generate the simulation track of color transition [21]. Color transition is different from ordinary morphing. It is constrained. What we use to demonstrate is traditional Chinese painting, which implies that all colors on the color transition track should be colors (as shown in Figure 9).

## 4. Experimental Analysis

In order to test the feasibility of the designed teaching system, simulate a Chinese painting with fading and halo as the experimental object, use the designed system and the original teaching system to teach the color of the Chinese painting, respectively, analyze the two groups of experimental data, and draw the experimental test conclusion [22].

We build the simulation experiment platform and set the experimental environment parameters. In order to ensure the accuracy of the two groups of experimental test results, simulate a color space, take the above color space as the color reference data to test the teaching effect, and use the two teaching systems to teach the color of Chinese painting. In this experiment, through the obtained painting scanning results, the recognition ability of the two teaching systems to the color halo or faded edge is analyzed.

### 4.1. Result Analysis

The experimental test results of the designed system are included in the experimental group. The test results of the original system are included in the reference group, the differences between the two groups are compared, the recognition ability of the teaching system is analyzed, and the experimental conclusion is drawn. According to the test results, the designed teaching system recognizes all the edges of the experimental object to form a closed edge curve. The system realizes the color teaching according to the closed edge to ensure that the color halo will not appear in the area after teaching. The original teaching system has a weak ability to identify the transition edge of painting color, resulting in the loss and jitter of the identified edge. At the same time, the edge line also has breakpoints, including some false edges, resulting in a large area of halo in the area taught according to the edge line, which is very different from the original color [23]. In order to further verify the teaching effect of Chinese painting color of the designed system, the intelligibility and fidelity of Chinese painting color are used as the effective measurement index of the teaching effect of the system. Through the color error analysis between the Chinese painting after teaching and the original image, the image quality is quantitatively evaluated. The Chinese painting with good quality has less error, higher understanding and fidelity, and higher similarity with the original image.

The deviation error between the traditional Chinese painting image after systematic teaching and the original image is used to objectively evaluate the quality of traditional Chinese painting after color teaching. The quality of traditional Chinese painting image is usually evaluated by time, mean square error, peak signal-to-noise ratio, or structural similarity.

Let the image size be *M* × *N*, the original image is represented by *I*_0_(*i*, *j*), and the image after teaching is represented by *I*_1_(*i*, *j*). The mean square error (MSE) of image quality evaluation after system teaching is as follows:

(7) $$\begin{array}{c} \text{MSE}=\frac{{\sum_{i=1}^{M}\sum_{j=1}^{N}\left[I_{0}\left(i,j\right)-I_{1}\left(i,j\right)\right]}^{2}}{M\times N}. \end{array}$$

In the formula, the smaller the value of MSE, the higher the quality of image teaching. The peak signal-to-noise ratio (PSNR) is as follows:

(8) $$\begin{array}{c} \text{PSNR}=10\times \mathrm{lg}\left(\frac{R^{2}}{MSE}\right). \end{array}$$

The higher the PSNR value, the better the image quality after teaching.

Combined with the similarity measurement results of all colors of Chinese painting, the final SSIM value of Chinese painting image is obtained. The larger the SSIM value, the better the image quality after teaching. We compare the execution time, mean square error, peak signal-to-noise ratio, and structural similarity of the two systems for color halo teaching and fading edge teaching in Chinese painting color teaching [24], and we evaluate the image quality of Chinese painting after the teaching of the two systems. The results are shown in Tables 1–5.

The comparison of the above experimental execution time and effect parameters is shown in Table 2.

By analyzing the data in Tables 1–5, it can be seen that the execution time of Chinese painting color teaching of the designed teaching system is far less than that of the original system. Among them, the execution time of image fading edge teaching is saved, which is 16.09 s shorter than that of the original system, which greatly improves the operation efficiency of the system. The mean square error of the designed teaching system is only about 50% of the original system, which greatly improves the sensory effect after image teaching, and the PSNR and SSIM of the designed teaching system are greater than the original system [25].

Figure 10 results show that the image quality of Chinese painting after the teaching of the designed system is higher and it is easier to achieve people's visual and ideal psychological recognition. From the above experimental results, compared with the Criminisi algorithm and the literature algorithm, the improved Criminisi algorithm proposed in this topic consumes relatively less time. The visual effect of teaching also meets the evaluation requirements, which verifies that the performance of the improved algorithm of this subject has been greatly improved and the teaching effect has been greatly improved when compared with other algorithms.

## 5. Conclusion

This paper presents an image reconstruction method based on 3D virtual reality technology. The experimental results show that the image reconstruction method based on 3D virtual reality technology has effectively improved the quality of the reconstructed image compared with the traditional image reconstruction method. In the environment based on differential sensitivity, the recall and precision of image pixel features are as high as 0.99. When reconstructing the noisy image, the peak signal-to-noise ratio and the standard signal-to-noise ratio of the reconstructed image by this method are higher than those based on very sparse random projection and sub-Gaussian random projection, which verifies the application value of this method. The systematic emphasis on splitting the concept of teaching object is based on the consideration of teaching feasibility, which is not completely consistent with the actual painting process. Moreover, because of the difficulty of extracting and describing teaching knowledge and the complexity of mural image content, it will take a long time to develop some image processing algorithms of all white movement. Not all the results produced by the system are satisfactory, and there are many human-computer interactions. This needs to continue to improve the whiteness and accuracy of a series of algorithms, such as automatic layering and region extraction, so as to facilitate and save the time of teaching a mural. Because of the difficulty of extracting and describing teaching knowledge and the complexity of mural image content, future research will focus on improving the automation and accuracy of image processing methods and minimizing human-computer interaction. This needs to continue to tap the deep knowledge of the field, continuously accumulate the chemical knowledge, empirical knowledge, and class library materials referred to in teaching, deeply study various color spaces, and improve a series of algorithms, such as automatic layering and region extraction.

Color teaching is an important part of Chinese painting teaching. In order to ensure that students learn color knowledge well, we need to let students master the spiritual connotation of color and fully apply it to color painting. Therefore, teachers need to pay attention to the transmission of spiritual connotation in color teaching and let students pay attention to and master its spiritual connotation through various effective ways, so as to improve students' ability to understand the color of Chinese painting and improve learning efficiency.

## Figures and Tables

**Figure 1:** Image color processing technology.

**Figure 2:** Relationship between computer graphics and related disciplines.

**Figure 3:** Basic model of image processing.

**Figure 4:** The mathematical model of image teaching problem.

**Figure 5:** Problems in continuous priority treatment of strong edges. The original image (a), mark the patched area (b), and the result image (c).

**Figure 6:** Normalization process of the image object.

**Figure 7:** Flowchart of color processing.

**Figure 8:** Three-dimensional analysis of traditional Chinese painting.

**Figure 9:** Color transition trajectory.

**Figure 10:** Monitoring error results.

**Table 1:** Evaluation results of Chinese painting image quality after two kinds of system teaching.

Quality evaluation index		Experience group	Test group
Execution time	Color halo teaching	16.38	26.35
	Fading edge teaching	16.35	29.36

MSE	Color halo teaching	2.39	6.58
	Fading edge teaching	3.68	6.35

PSNR	Color halo teaching	31.39	29.38
	Fading edge teaching	26.38	29.58

SSIM	Color halo teaching	0.8963	0.9687
	Fading edge teaching	0.9632	0.9541

**Table 2:** Comparison of execution time of two algorithms.

Mural image to be taught	Time taken by Criminisi algorithm (seconds)	The time taken by the algorithm of this subject (seconds)
Experimental mural I	26.35	16.38
Experimental mural 2	24.39	18.36
Experimental mural 3	29.36	25.36

**Table 3:** Comparison of PSNR effects of three teaching algorithms.

PSNR (dB)			
	Experimental mural 1	Experimental mural 2	Experimental mural 3
Criminisi algorithm	25.39	26.38	29.54
Literature algorithm	24.36	27.12	31.68
Algorithm of this subject	29.58	27.58	32.68

**Table 4:** Comparison of SSIM effects of three teaching algorithms.

SSIM			
	Experimental mural 1	Experimental mural 2	Experimental mural 3
Criminisi algorithm	0.9563	0.9423	0.9521
Literature algorithm	0.9452	0.9432	0.9534
Algorithm of this subject	0.9231	0.9874	0.9581

**Table 5:** Comparison of the monitoring error results of the three teaching algorithms.

Monitoring error results		
	The first group of experiments	The second group of experiments
Criminisi algorithm	20.3%	38.3%
Literature algorithm	17.3%	26.4%
Algorithm of this subject	8.6%	16.5%

## Data Availability

The labeled dataset used to support the findings of this study is available from the corresponding author upon request.
